The article "Relationships among Coracobrachialis, Biceps Brachii, and Pectoralis Minor Muscles and Their Correlation with Bifurcated Coracoid Process" was published in 2022. Journal: Biomed Res Int.

# Relationships among Coracobrachialis, Biceps Brachii, and Pectoralis Minor Muscles and Their Correlation with Bifurcated Coracoid Process

**DOI:** 10.1155/2022/8939359

**Published:** 2022-03-25

**Authors:** Nicol Zielinska, R. Shane Tubbs, Michał Podgórski, Marko Konschake, Paloma Aragonés, Dariusz Grzelecki, Łukasz Olewnik

**Affiliations:** ^1^Department of Anatomical Dissection and Donation, Medical University of Łódź, Poland; ^2^Department of Neurosurgery, Tulane University School of Medicine, New Orleans, LA, USA; ^3^Department of Neurosurgery and Ochsner Neuroscience Institute, Ochsner Health System, New Orleans, LA, USA; ^4^Department of Anatomical Sciences, St. George's University, Grenada; ^5^Department of Neurology, Tulane University School of Medicine, New Orleans, LA, USA; ^6^Department of Structural and Cellular Biology, Tulane University School of Medicine, New Orleans, LA, USA; ^7^Department of Diagnostic Imaging, Polish Mother's Memorial Hospital-Research Institute, Łódź, Poland; ^8^Institute of Clinical and Functional Anatomy, Medical University of Innsbruck (MUI), Innsbruck, Austria; ^9^Department of Orthopedics Surgery, Hospital Santa Cristina, Madrid, Spain; ^10^Department of Human Anatomy and Embryology, Facultad de Medicina, Universidad Complutense de Madrid, Spain; ^11^Department of Orthopedics and Rheumoorthopedics, Centre of Postgraduate Medical Education, Otwock, Poland

## Abstract

The aim of this study is to demonstrate the relationship between the proximal attachment of the coracobrachialis muscle and the short head of the biceps brachii and the distal attachment of the pectoralis minor. Their correlation with the bifurcated coracoid process (CP) will be also assessed. On the basis of these observations, a new classification of structures attached to the coracoid process is proposed. Classical anatomical dissection was performed on one hundred forty-five upper limbs. Three types of relationship between the coracobrachialis muscle and the short head of the biceps brachii were observed in the cadavers. In type I (occurring in 54%), the coracobrachialis and the short head of the biceps brachii created a common junction attached to a single CP. Type II was divided into two subtypes (a and b). Subtype IIa (frequency 10%) was represented by independent proximal attachments of the short head of the biceps brachii and the coracobrachialis muscles to the CP. In subtype IIb (frequency 5%), the coracobrachialis muscle was two-headed (the first head located under the second) and not connected to the short head of the biceps brachii; all heads were attached to a single CP. Type III (frequency 31%) was characterized by a two-headed coracobrachialis muscle, the first head originating from a bifurcated CP laterally to the short head of the biceps brachii and the second medially to this structure. Different variations connected with the mentioned structures could be problematic for surgeons during operations, so detailed knowledge of them could contribute to more efficient procedures.

## 1. Introduction

The anterior compartment of the arm consists of the biceps brachii muscle (BB), the coracobrachialis muscle (CBM), and the brachialis muscle. The BB has two heads: a long head (lhBB) originating from the supraglenoid tubercle and a short head (shBB) originating from the apex of the coracoid process (CP) of the scapula. In most cases, this creates a common junction with the proximal attachment of the CBM [1]. Both the CBM and shBB function in adduction of the arm [2, 3]. Another muscle responsible for the same movement is the pectoralis minor (PM) [4]. This is also attached to the CP. Branches arising from the brachial artery supply blood to the CBM and shBB, and the musculocutaneous nerve innervates these structures [5]. The PM is supplied by the thoracoacromial artery (a branch of the axillary artery) and innervated by the lateral and medial pectoral nerves [6].

As mentioned above, a common function of these three muscles is adduction of the arm at the glenohumeral joint [2, 3, 7]. They also have other functions. For example, the BB is responsible for flexion of the elbow and supination of the forearm, the CBM is a flexor of the arm, and the PM is an accessory inspiratory muscle [8, 9].

Morphologically, they are variable [3, 8, 10–15]. Some variations are connected with some kind of additional structure. For instance, there are descriptions in the available literature of a CBM with four [8] or even six [16] heads, and the BB with five heads [12]. Proximal or distal attachments sites can also differ [5]. There are cases featuring an accessory muscle connected with one of these muscles, such as the coracobrachialis superior [17], the coracobrachialis longus [15], or the accessory pectoralis muscle [18].

In most cases, additional structures such as heads or accessory muscles correlate with some kind of neurovascular compression [15]. One example is compression of the musculocutaneous nerve (MCN) when it courses between two CBM heads [15]. In some situations, the PM can cause subclavicular brachial plexus compression, potentially leading to pectoralis minor syndrome [19]. An additional head of the BB can result in median nerve entrapment, thrombosis, or edema [20]. Of course, morphological variations are not only related to such conditions. Importantly, any morphological variation can be problematic for the surgeon, so detailed knowledge of possible morphological variabilities seems indispensable for a qualified specialist [21].

The aim of this study is to examine the statistical significance of the relationship between the morphometric features of the proximal attachments of the coracobrachialis and BB, and the distal attachment of the pectoralis minor muscle, and their correlation with a bifurcated CP. Another related aim is to create a new classification of structures attached to the CP. The CP is also characterized as single or bifurcated. To our knowledge, this is the first such study.

## 2. Materials and Methods

One hundred forty-five upper limbs were examined (99 from females with mean age at death 81.4 years ± 12.2 and 46 males with mean age at death 78.1 years ± 12.0; 73 right and 72 left arms, fixed in 10% formalin). The cadavers were the property of the Department of Anatomical Dissection and Donation of the Medical University of Łódź, Poland, and of the Donors and Dissecting Rooms Center, Universidad Complutense de Madrid, Spain, following donations to the university anatomy programs. Any upper limbs with evidence of surgical intervention in the dissected area were excluded and were not counted among the limbs examined. All dissections of the shoulder and arm areas were performed following preestablished protocols [5, 8, 22–26].

Dissection began with removal of the skin and superficial fascia from the area of the shoulder and the anteromedial side of the arm and the anterior side of the forearm. The next step included visualizing the lateral, medial, and posterior cords of the brachial plexus and accurate visualization of the brachialis muscle, the CBM, and the shBB. The muscle belly was thoroughly cleaned, and the tendons or tendon was cleaned and checked in the proximal direction. The distal attachment of the PM was then visualized. Possible additional structures such as accessory heads were recorded. Following this, all structures were thoroughly cleaned. Upon dissection, the following morphological features were assessed:

- The number of heads of the CBM
- The location of the proximal attachments of the CBM and shBB and the distal attachment of the PM
- Morphometric measurements (width, thickness, and length) of the shBB, the CBM, and the PM
- Type of CP

### 2.1. Statistical Analysis

Statistica 13.1 was used (Dell Inc. (2016), Dell Statistica (data analysis software system), version 13. http://software.dell.com/.). A *p* value lower than 0.05 was considered significant; a Bonferroni correction was used for multiple testing.

The chi-square test was used to compare differences between sex/side and among specimens in attachments of the shBB, the CBM, and the PM located on the CP. It was also applied to check differences in the presence of a capsular band between attachment types.

For the analysis of continuous variables, the Shapiro-Wilk test was used first to assess the normality of the data distribution. Since the distribution was other than normal in all variables compared, nonparametric tests were used:

- The Mann-Whitney for comparing morphological data between sexes and coracoid process types
- The Wilcoxon sign rank test for comparing morphological data between sides when both limbs were from the same donor
- The Kruskal-Wallis test by ranks with dedicated post hoc test for comparing morphological data between different types of origin

## 3. Results

The cadaveric material comprised 145 upper limbs. In only three cases were limbs from separate specimens; the remaining 142 were obtained as pairs from the same cadaver.

The first field of variation concerned the origin of the shBB and the coracobrachialis muscles. The following types were differentiated morphologically (F, females; M, males; R right limb; L, left limb):

(i) Type I: characterized by one head of the CBM and the shBB creating a common junction originating from the CP. The frequency was 54% (58 F and 21 M; 40 R and 39 L) (Figure 1)
(ii) Type II: characterized by independent attachment of the CBM and shBB originating from the CP. The frequency was 15% (13 F and 10 M; 11 R and 12 L)
  - Subtype IIa: independent proximal attachments of one-headed CBM and the shBB originating from the CP. The frequency was 10% (eight F and six M; seven R and seven L) (Figure 2)
  - Subtype IIb: independent two-headed CBM (the first head located under the second), not connected to the shBB, originating from the CP. The frequency was 5% (five F and four M; four R and five L) (Figures 3 and 4)
(iii) Type III: characterized by two-headed CBM: the first originating from the CP laterally to the shBB and the second medially to this structure. The frequency was 31% (30 F and 15 M; 24 R and 21 L) (Figure 5)

In the region of the CP, we observed two main types of anatomical variation. The first concerned the shape of the CP itself. It was single or bifid.

- Type 1: characterized by a single CP. The frequency was 69% (71 F and 31 M; 51 R and 51 L)
- Type 2: characterized by a bifid CP. The frequency was 30% (28 F and 15 M; 24 R and 21 L)

There were no significant differences between sexes (*p* = 0.0849) or body sides (*p* = 0.5685) in the two types of process.

Only the type III relationship between shBB and CBM cooccurred with the bifid CP (*p* = 0.0001).

The comparisons of morphological data between sexes and body sides are presented in Table 1; the origins and CP types are compared in Table 2.

According to post hoc analysis, the short head belly was significantly longer in type 2 than type 1 origins. The coracobrachialis 1/medial and 2/lateral were significantly shorter in the type 1 origin than the two other types.

Interestingly, in a single type of CP and in types 1 and 2 short head origins, we found an additional band from the short head tendon attaching to the capsule of the glenohumeral joint. It was present in 12 cases (only in females, *p* = 0.0334; six L and six R, *p* = 0.9412). Its mean length was 13.61 ± 1.75 mm. Its proximal width and thickness were 4.10 ± 0.82 mm and 1.73 ± 0.55 mm, respectively; its distal width and thickness were 4.90 ± 0.87 mm and 2.15 ± 0.61 mm, respectively. There were no significant differences in these morphological parameters between types of short head origin.

## 4. Discussion

The main value of the work is its presentation of the relationship between the CBM, the shBB, and the PM, taking into consideration the morphometric measurements of their attachments to the CP, the type of CP (single or bifurcated), and features such as the number of bellies. It should be emphasized that this is the first study of such a relationship and it could be of value for orthopedists and surgeons operating in this area. It could also be useful for physiotherapists planning rehabilitation procedures and radiologists interpreting images. Rigid anatomical norm included in classical textbooks may create an overgeneralized image of the human body that is not always true in reality. Hence, there is a need to reproduce known anatomical research based on the dissection of a large sample [27].

Our results suggested a new classification system based on the relationship between the shBB and CBM. Type I was characterized by one head of the CBM and the shBB, creating a common junction originating from the CP. This was the most common type. Type II, characterized by independent attachments of the CBM and shBB originating from the CP, was divided into two subtypes. The first was represented by one head of the CBM and the second by two, one of which was located under the other. Type III was characterized by a two-headed CBM: the first originating from the CP laterally to the shBB and the second medially to this structure.

An additional head of the CBM could predispose to neurovascular compression, for example, of the MCN, which in some cases courses between two CBM heads. In our study, subtype IIb and type III were represented by two-headed CBMs, so these types are probably associated with weakness of the anterior compartment of the arm, resulting in problems in flexion and abduction in the glenohumeral joint. The MCN also provides sensory innervation to the elbow joint and the lateral part below the elbow joint to the distal parts of the fingers. It is associated with tingling or numbness.

The next question concerns the possible clinical significance of differences between the proximal attachments of the shBB and CBM with a common junction and proximal attachments with two distinct origins. We hypothesize that the common junction (type I) increases the strength of these two muscles. On the other hand, a division between the proximal parts of the shBB and CBM (subtype IIa) could indicate reduced strength but also the possibility of more complex movements. Hypothetically, therefore, type I predisposes to greater strength, but subtype II allows for more precise movements.

The structure of the CP was also assessed, and the results suggested two types, single and bifurcated. Interestingly, the bifurcated CP correlated only with type III, characterized by one head of the CBM located laterally to the shBB and the second located medially to it. In our opinion there are two possibilities. First, the split CP is the main morphological variation, and the type III presentation of the shBB and CBM is a result of this divided CP. Second, the relationship between the shBB and the two heads of the CBM assessed as type III is the main variation, and the split CP is an adaptation to this type.

A study of embryogenesis will help us to evaluate these hypotheses. There are two possibilities for embryogenesis of the CP. The divided CP could arise from displacement of one of the ossification centers during intrauterine growth. Alternatively, it could arise from more than two ossification centers, one of which participates in creating an additional structure. It is also possible that during early embryogenesis, the CP is single and then it starts to form a broad base, splitting from the center into two parts [28]. It is worth mentioning that ossification of the CP generally starts 3-4 months after birth, though sometimes it begins before birth. However, it continues; the center of ossification expands and creates a region of true bipolar growth between the CP and the main part of the scapula up to the age of two [29]. In 1974, it was determined that the cause of the split CP could be an ontogenic mishap, its onset preceding chondrification of the scapular anlage [30].

The above information shows that formation of the CP is a long process, but we should also consider the embryogenesis of the CBM. This begins with derivation from a common premuscle mass derived from the lateral mesoderm. This process is characteristic not only of the CBM but also of the BB and the PM, so these three structures are closely connected. The premuscle mass then regresses, and division into three distinct muscles ensues. This process should end when the embryos reach 14-16 mm in length [31]. The situation when the CBM is represented by two heads, one originating laterally and the other medially to the shBB, could be the result of wrong or premature termination of this division into three muscles.

Summing up the foregoing, embryogenesis of the CBM should end during pregnancy. The development of the CP is a complex process, and complete shaping of this structure continues for two years after birth. We can therefore infer that the divided CP is something like an adaptation for type III characterized by one head of the CBM being located lateral to the shBB and the second medial. It sounds logical; but what is the mechanism of this adaptation?

Normally, the origin of the CBM is medial to that of the shBB, and they usually create a common junction. Their main function is adduction of the arm. On the other hand, the long head of the biceps brachii muscle (lhBB), located laterally to the shBB, is responsible for abduction of the arm. Of course, the lhBB is attached to the supraglenoid tubercle, but some explanation could be found. Both heads of the CBM are located on the CP, but hypothetically, its lateral head could be more involved during abduction and less during adduction than its medial head. The lateral head of the CBM could then generate an expansion force resulting in a lateral bulge on the CP. The same is true for the second head, which could generate an expansion force resulting in a medial bulge on the CP. The shBB is located between these two structures, so it could act as a stabilizer of the CP, and thanks to this a small recess could be created between the two bulges.

The proposed process seems difficult to implement in a mature bone structure. The CP is more likely to suffer microinjuries, so in old age, it would become more susceptible to degeneration. However, the most important thing is that the center of ossification of the CP expands and produces a true bipolar growth region up to the age of two.

Children after birth make many arm movements a day. So, if their course of the CBM and shBB is the same as in type III, the CP is constantly exposed to the expansion forces. Ossification continues and the forces described are involved in forming the CP. Of course, as mentioned above, this is only our hypothesis, but it seems likely to be the main cause of the split CP, which cooccurred only with type III.

Our statistical results could also help to identify the adaptive change. If not all cases represented by type III were connected with a split CP, we would conclude that this type of CP was created for adaptation, which did not occur in all cases. If the split CP cooccurred with other types as well as type III, we would conclude that such a specific presentation of type III was more likely to indicate an adaptive change.

However, our statistical results cannot be helpful because every type III case (one head of the CBM located laterally to the shBB and the second located medially) had a split CP. The split CP and type III occurred in 45 cases (30 female and 15 male), more specifically in 24 right and 21 left upper limbs, making the frequency 31% of the studied population.

Knowledge of morphological variations of this region could also be clinically useful. Recurrent anterior glenohumeral instability is a common disorder among patients who are young, male, and active and have bone defects or ligament laxity [32]. One method used to treat it is the Latarjet procedure, which involves transfer of the osteomized CP (together with tendons attached to this structure, the shBB and CBM) to the anterior glenoid [33]. This procedure involves making an incision along the anterior axillary line and transection of the coracoacromial ligament laterally to the CP (for hassle-free repair of the anterior capsule). The next stage depends on the release of the PM subperiosteally from the medial part of the CP and transection of the CP medially to laterally. A longitudinal capsulotomy should follow. The capsule and labrum are removed from the anterior aspect of the glenoid. The next stage depends on attachment of the part of the CP to this region [28]. This procedure should end with repair of the intersected structures and tissues [34].

Type III stands out in this situation, too. As mentioned above, it was connected with the bifurcated CP in all cases. How would this affect the procedure? Hypothetically, it is possible to use only the lateral part of the CP to transfer it to the anterior glenoid. This seems less invasive because the shBB and the medial head of the CBM are not connected to this region of the CP, so the incision or transferring of these structures with a fragment of the CP could be unnecessary.

Type IIb, characterized by an independent shBB and two heads of the CBM (the first attached laterally to the shBB and the second located under these two structures), could entail a more complicated operation. An extra head of the CBM revealed by computed tomography or magnetic resonance could confuse a surgeon. It is even worse if the change is detected during an operation. Complications or prolongation of the surgery could result [21].

Another morphological variation is an additional band from the shBB attaching to the capsule of the glenohumeral joint. In our study, this structure occurred in only 12 cases (8%). However, such a variation could also confuse a surgeon and make surgery more difficult.

Anatomical variations of the biceps brachii and coracobrachialis muscles may occasionally be accompanied by an atypical course of nerves or arteries [35, 36].

The present study has some limitations. First, a larger sample size would have been desirable; however, the small size (*n* = 145) was a consequence of the muscles' morphological variability. Secondly, the study population was recruited from a specific group of people who had lived the better part of their lives around Łódź, Poland, and Madrid, Spain. More extensive studies on wider populations are needed. Nevertheless, our study is the first of this magnitude to propose a new classification based on the relationship between the origins of the CBM and shBB.

Summing up, knowledge of the various types of these muscles could be useful in the Latarjet procedure. Every type characterized by occurrence of the additional structure, such as an extra head or band from the shBB, which is a rare element, could make the operation more problematic. On the other hand, type III could in our opinion predispose to a less invasive procedure; so, as in any situation, there are pros and cons.

Development of the CP and the CBM could suggest that the split CP is an adaptive change for the two-headed CBM, one head attached laterally to the shBB and the other medially. To test this hypothesis, more embryogenetic studies are needed.

## 5. Conclusion

The relationship between the origins of the CBM and shBB is variable. The most distinctive variant is type III, the only one that cooccurred with the split CP. Analyzing their embryogenesis and postnatal development, we concluded that the split CP was most likely to be the adaptive change, not the other way around. Different variations connected with the mentioned structures can be problematic for surgeons during operations, so detailed knowledge of them can lead to more efficient procedures. The morphological features of the PM showed no statistical significance.

## Figures and Tables

**Figure 1:** Type I. CP: coracoid process; PMM: pectoralis minor muscle; DM: deltoid muscle; CBM: coracobrachialis muscle; shBB: short head of the biceps brachii; lhBB: long head of the biceps brachii.

**Figure 2:** Type IIa. CP: coracoid process; DM: deltoid muscle; CBM: coracobrachialis muscle; shBB: short head of the biceps brachii; lhBB: long head of the biceps brachii; H: humerus; LC: lateral cord of the brachial plexus; MCN: musculocutaneous nerve; SSM: subscapularis muscle.

**Figure 3:** Type IIb. CP: coracoid process; DM: deltoid muscle; CBM: coracobrachialis muscle; shBB: short head of the biceps brachii; lhBB: long head of the biceps brachii; H: humerus.

**Figure 4:** Type IIb with cut-off anatomical structures of the proximal attachment. The purple-dotted circles indicates both independent head of the coracobrachialis muscle, while the green-dotted line indicates cut-off short head of the biceps brachii. CP: coracoid process; DM: deltoid muscle; CBM: coracobrachialis muscle; shBB: short head of the biceps brachii; lhBB: long head of the biceps brachii.

**Figure 5:** Type III. CP: coracoid process; PMM: pectoralis minor muscle; DM: deltoid muscle; CBM: coracobrachialis muscle; shBB: short head of the biceps brachii; lhBB: long head of the biceps brachii; H: humerus.

**Table 1:** Morphometric parameters according to sex and body side. All data are presented in millimeters.

Parameter		Sex		*p* value	Body side		*p* value
		Females	Males		Right	Left	
Pectoralis muscle	Width	11.63 (3.30)	13.84 (3.83)	0.0015∗	12.63 (3.64)	12.00 (3.58)	0.3929
	Thickness	2.78 (1.02)	2.92 (1.08)	0.5419	2.91 (1.08)	2.74 (0.99)	0.2946

Coracoid—short head	Width	11.91 (3.71)	13.04 (3.91)	0.2793	12.39 (3.65)	12.02 (3.93)	0.7874
	Thickness	3.25 (1.24)	3.73 (1.02)	0.0563	3.43 (1.19)	3.33 (1.22)	0.7649

Coracobrachialis 1/medial	Width	7.87 (2.14)	8.77 (2.63)	0.1356	8.28 (2.19)	8.14 (2.55)	0.7825
	Thickness	2.50 (0.79)	2.99 (1.02)	0.1468	2.63 (0.92)	2.74 (0.90)	0.5498

Coracobrachialis 2/lateral	Width	9.82 (3.87)	7.63 (4.10)	0.1388	8.71 (4.14)	9.08 (4.09)	0.8738
	Thickness	3.14 (1.71)	2.24 (0.71)	0.0062	2.83 (1.77)	2.67 (0.98)	0.8567

Short head of biceps brachii	Width	6.76 (2.16)	6.77 (1.64)	0.8041	6.64 (1.97)	6.89 (2.00)	0.6498
	Thickness	2.06 (0.63)	2.38 (0.85)	0.0451	2.17 (0.70)	2.19 (0.77)	1.0000
	Tendon length	75.83 (19.66)	78.98 (20.77)	0.2665	78.65 (18.68)	74.90 (21.23)	0.3356
	Belly length	159.34 (18.65)	166.35 (21.82)	0.0009∗	158.81 (20.61)	164.30 (18.91)	0.1469

Myotendinous junction	Width	8.48 (2.86)	9.01 (2.47)	0.1535	8.32 (2.64)	9.00 (2.83)	0.1455
	Thickness	3.18 (1.21)	3.79 (1.83)	0.0118	3.27 (1.01)	3.48 (1.81)	0.9621

Coracobrachialis 1/medial length		117.90 (20.57)	126.41 (21.32)	0.0376	121.80 (18.25)	119.35 (23.80)	0.7145
Coracobrachialis 2/lateral length		102.70 (25.86)	111.89 (32.82)	0.0235	104.62 (30.26)	108.35 (27.71)	0.6266
Coracobrachialis 3 length		49.14 (16.30)	65.21 (33.97)	0.5309	56.57 (27.35)	57.78 (28.85)	1.0000

Level of significance level according to the Bonferroni correction was 0.003 and marked with ∗.

**Table 2:** Morphometric parameters according to insertion type. All data are presented in millimeters.

Parameter		Origin type			*p*	Coracoid process		*p*
		I	II	III		Single	Bifid	
Pectoralis muscle	Width	11.56 (3.14)	12.80 (4.83)	13.42 (3.42)	0.0103	11.84 (3.60)	13.42 (3.42)	0.0058
	Thickness	2.86 (1.06)	2.81 (0.95)	2.76 (1.05)	0.7359	2.85 (1.03)	2.76 (1.05)	0.4393

Coracoid—short head	Width	12.21 (3.77)			—	12.21 (3.77)		—
	Thickness	3.38 (1.20)			—	3.38 (1.20)		—

Coracobrachialis 1/medial	Width	8.21 (3.22)	8.69 (2.55)	7.97 (2.23)	0.5407	8.64 (2.57)	7.97 (2.23)	0.2827
	Thickness	3.40 (0.51)	2.80 (1.03)	2.58 (0.85)	0.1083	2.87 (1.00)	2.58 (0.85)	0.1179

Coracobrachialis 2/lateral	Width	6.25 (2.43)	10.39 (3.47)	8.63 (4.25)	0.3249	9.61 (3.63)	8.63 (4.25)	0.5772
	Thickness	2.38 (0.82)	3.03 (0.95)	2.70 (1.59)	0.2286	2.91 (0.94)	2.70 (1.59)	0.1762

Short head of biceps brachii	Width		6.11 (1.56)	7.10 (2.09)	0.1558	6.11 (1.56)	7.10 (2.09)	0.1558
	Thickness		2.05 (0.80)	2.24 (0.69)	0.2649	2.05 (0.80)	2.24 (0.69)	0.2649
	Tendon length	76.46 (21.89)	69.76 (17.61)	81.04 (16.64)	0.0604	74.95 (21.11)	81.04 (16.64)	0.0856
	Belly length	157.55 (19.23)	171.56 (19.63)	165.08 (19.27)	0.0028∗	160.49 (20.05)	165.08 (19.27)	0.1469

Myotendinous junction	Width	8.90 (3.00)	7.76 (2.21)	8.62 (2.45)	0.3269	8.66 (2.88)	8.62 (2.45)	0.9149
	Thickness	3.47 (1.73)	2.93 (1.43)	3.41 (0.80)	0.0290	3.35 (1.67)	3.41 (0.80)	0.0696

Coracobrachialis 1/medial length		114.43 (21.78)	129.87 (23.41)	127.11 (14.70)	0.0007∗	127.11 (14.70)	117.67 (22.90)	0.0073
Coracobrachialis 2/lateral length		71.20 (38.87)	109.67 (24.82)	117.11 (13.44)	0.0001∗	89.06 (37.94)	117.11 (13.44)	0.0010∗
Coracobrachialis 3 length		55.94 (29.83)		62.13 (6.00)	0.5139	55.94 (29.83)	62.13 (6.00)	0.5139

Level of significance level according to the Bonferroni correction was 0.003 and marked with ∗.

## Data Availability

Please contact the author for data requests (Łukasz Olewnik, PhD—email address: lukasz.olewnik@umed.lodz.pl).

## References

[1] Moore K. L., Dalley A. F. (2013). Clinically oriented anatomy.

[2] El-Naggar M. M., Al-Saggaf S. (2004). Variant of the coracobrachialis muscle with a tunnel for the median nerve and brachial artery. *Clinical Anatomy*.

[3] Georgiev G. P., Tubbs R. S., Landzhov B. (2018). Coracobrachialis longus muscle: humeroepitrochlearis. *Cureus*.

[4] Morais N., Cruz J. (2016). The pectoralis minor muscle and shoulder movement-related impairments and pain: rationale, assessment and management. *Physical Therapy in Sport*.

[5] Szewczyk B., Polguj M., Paulsen F. (2021). A proposal for a new classification of coracobrachialis muscle morphology. *Surgical and Radiologic Anatomy*.

[6] Moriya A., Takafuji T., Sato Y. (1993). Arterial supply in the human pectoralis minor muscle. *Okajimas Folia Anatomica Japonica*.

[7] Baig M. A., Bordoni B. (2019). *Anatomy, Shoulder and Upper Limb, Pectoral Muscles*.

[8] Olewnik Ł., Zielinska N., Karauda P., Duparc F., Georgiev G. P., Polguj M. (2021). The co-occurrence of a four-headed coracobrachialis muscle, split coracoid process and tunnel for the median and musculocutaneous nerves: the potential clinical relevance of a very rare variation. *Surgical and Radiologic Anatomy*.

[9] Podgórski M., Olewnik Ł., Rusinek M., Cichosz M., Polguj M., Topol M. (2019). ‘Superior biceps aponeurosis’—morphological characteristics of the origin of the short head of the biceps brachii muscle. *Annals of Anatomy-Anatomischer Anzeiger*.

[10] Ballesteros L. E., Forero P. L., Buitrago E. R. (2014). Evaluation of additional head of biceps brachii: a study with autopsy material. *Folia Morphologica*.

[11] Greig H., Anson B., Budinger J. (1952). Variations in the form and attachments of the biceps brachii muscle. *Quarterly Bulletin of Northwestern University Medical School*.

[12] Je S. S., Park B., Kim J., Yoon S. P. (2016). Five-headed biceps brachii muscle with a rare origin from the tendon of pectoralis major muscle. *Anatomical Science International*.

[13] Kopuz C., Sancak B., Özbenli E. (1999). On the incidence of third head of biceps brachii in Turkish neonates and adults. *Kaibogaku zasshi. Journal of Anatomy*.

[14] Kosugi K., Shibata S., Yamashita H. (1992). Supernumerary head of biceps brachii and branching pattern of the musculocutaneus nerve in Japanese. *Surgical and Radiologic Anatomy*.

[15] Olewnik P. F., Tubbs R. S., Zielinska N., Szewczyk B., Karauda P., Polguj M. (2021). Potential compression of the musculocutaneous, median and ulnar nerves by a very rare variant of the coracobrachialis longus muscle. *Folia Morphologica*.

[16] Zielinska N., Olewnik Ł. (2021). Six-headed coracobrachialis muscle. *Folia Morphologica*.

[17] Olewnik Ł., Zielinska N., Gołek Ł., Aragonés P., Sanudo J. R. (2021). Is it the coracobrachialis superior muscle, or is it an unidentified rare variant of coracobrachialis muscle?. *Surgical and Radiologic Anatomy*.

[18] Bannur B. M., Mallashetty N., Endigeri P. (2013). An accessory muscle of pectoral region: a case report. *Journal of Clinical and Diagnostic Research: JCDR*.

[19] Sanders R. J., Rao N. M. (2010). The forgotten pectoralis minor syndrome: 100 operations for pectoralis minor syndrome alone or accompanied by neurogenic thoracic outlet syndrome. *Annals of Vascular Surgery*.

[20] Yershov D., Hudák R. (2015). Unusual variation of the biceps brachii with possible median nerve entrapment. *Prague Medical Report*.

[21] Kopuz C., Içten N., Yildirim M. (2003). A rare accessory coracobrachialis muscle : a review of the literature. *Surgical and Radiologic Anatomy*.

[22] Olewnik Ł., Karauda P., Gonera B. (2021). Impact of plantaris ligamentous tendon. *Scientific Reports*.

[23] Olewnik Ł., LaPrade R. F., Paulsen F. (2021). A proposal for a new morphological classification of the popliteus muscle tendon with potential clinical and biomechanical significance. *Scientific Reports*.

[24] Zielinska N., Olewnik Ł., Karauda P., Tubbs R. S., Polguj M. (2021). A very rare case of an accessory subscapularis muscle and its potential clinical significance. *Surgical and Radiologic Anatomy*.

[25] Zielinska N., Tubbs R. S., Borowski A., Podgórski M., Olewnik Ł. (2021). The subscapularis muscle: a proposed classification system. *BioMed Research International*.

[26] Zielinska N., Tubbs R. S., Podgórski M., Karauda P., Polguj M., Olewnik Ł. (2021). The subscapularis tendon: a proposed classification system. *Annals of Anatomy-Anatomischer Anzeiger*.

[27] Żytkowski A., Tubbs R. S., Iwanaga J., Clarke E., Polguj M., Wysiadecki G. (2021). Anatomical normality and variability: historical perspective and methodological considerations. *Translational Research in Anatomy*.

[28] Sharma B. G. (2003). Duplication of the clavicle with triplication of the coracoid process. *Skeletal Radiology*.

[29] Ogawa K., Inokuchi W., Matsumura N. (2020). Physeal injuries of the coracoid process are closely associated with sports activities: a systematic review. *Orthopaedic Journal of Sports Medicine*.

[30] McClure J. G., Raney R. B. (1974). Double acromion and coracoid processes. *The Journal of Bone and Joint Surgery. American Volume*.

[31] Olewnik Ł., Podgórski M., Ruzik K., Polguj M., Topol M. (2020). New classification of the distal attachment of the fibularis brevis — anatomical variations and potential clinical implications. *Foot and Ankle Surgery*.

[32] Woodmass J. M., Wagner E. R., Solberg M., Hunt T. J., Higgins L. D. (2019). Latarjet procedure for the treatment of anterior glenohumeral instability. *JBJS Essential Surgical Techniques*.

[33] Latarjet M. (1958). Technic of coracoid preglenoid arthroereisis in the treatment of recurrent dislocation of the shoulder. *Lyon Chirurgical*.

[34] Sharareh B., Edwards T. B., Shah A., Shybut T. (2021). Variation in technique and postoperative management of the Latarjet procedure among orthopedic surgeons. *Journal of Shoulder and Elbow Surgery*.

[35] Clarke E., Tubbs R. S., Radek M., Haładaj R., Tomaszewski M., Wysiadecki G. (2021). Unusual formation of the musculocutaneous and median nerves: a case report refined by intraneural dissection and literature review. *Folia Morphologica*.

[36] Zhou M., Ishizawa A., Akashi H., Suzuki R., Bando Y. (2021). Bilateral accessory heads of biceps brachii muscle coexisting with brachioradial artery passing between two layers of atypical bicipital aponeurosis. *Translational Research in Anatomy*.

[37] Iwanaga J., Singh V., Ohtsuka A. (2021). Acknowledging the use of human cadaveric tissues in research papers: recommendations from anatomical journal editors. *Clinical Anatomy*.

